# Diarrhea management in children under five in sub-Saharan Africa: does the source of care matter? A Countdown analysis

**DOI:** 10.1186/s12889-016-3475-1

**Published:** 2016-08-19

**Authors:** Liliana Carvajal-Vélez, Agbessi Amouzou, Jamie Perin, Abdoulaye Maïga, Hayalnesh Tarekegn, Akanni Akinyemi, Solomon Shiferaw, Mark Young, Jennifer Bryce, Holly Newby

**Affiliations:** 1 United Nations Children’s Fund UNICEF, 3 UN Plaza, New York City, NY 10017 USA; 2 Johns Hopkins University, International Health, Baltimore, USA; 3 Université catholique de Louvain, Louvain-la-Neuve, Belgium; 4 Obafemi Awolowo University, Ile Ife, Nigeria; 5 Addis Ababa University, School of Public Health, Addis Ababa, Ethiopia

**Keywords:** Child health, Diarrhea, Household surveys, Health providers, Oral rehydration salts

## Abstract

**Background:**

Diarrhea remains a high burden disease, responsible for nine percent of deaths in children under five globally. We analyzed diarrhea management practices in young children and their association with the source of care.

**Methods:**

We used Demographic and Health Survey data from 12 countries in sub-Saharan Africa with high burdens of childhood diarrhea. We classified the quality of diarrhea management practices as good, fair, or poor based on mothers’ reports for children with diarrhea, using WHO/UNICEF recommendations for appropriate treatment. We described the prevalence of diarrhea management by type and assessed the association between good management and source of care, adjusting for potential confounders.

**Results:**

Prevalence of good diarrhea management is low in 11 of the 12 analyzed surveys, varying from 17 % in Cote d’Ivoire to 38 % in Niger. The exception is Sierra Leone, where prevalence of good practice is 67 %. Prevalence of good management was low even among children taken to health facilities [median 52 %, range: 34–64 %]. Diarrhea careseeking from health facilities or community providers was associated with higher odds of good management than care from traditional/informal sources or no care. Careseeking from facilities did not result systematically in a higher likelihood of good diarrhea management than care from community providers. The odds of good diarrhea management were similar for community versus facility providers in six countries, higher in community than facility providers in two countries, and higher in facility than in community providers in four countries.

**Conclusion:**

Many children’s lives can be saved with correct management of childhood diarrhea. Too many children are not receiving adequate care for diarrhea in high-burden sub-Saharan African countries, even among those seen in health facilities. Redoubling efforts to increase careseeking and improve quality of care for childhood diarrhea in both health facilities and at community level is an urgent priority.

## Background

Diarrheal disease is highly preventable, yet accounts for nine percent of all deaths among children under age five worldwide [12]. In 2013, this translated into about 580,000 child deaths, or, on average, 1,600 children dying each day due to preventable diarrhea [21]. Most deaths from diarrhea occur among children less than 2 years of age living in South Asia and sub-Saharan Africa [9]. In 2004, WHO and UNICEF issued a joint statement on clinical treatment of acute diarrhea, recommending the use of low-osmolarity oral rehydration salts (ORS), zinc supplementation, increased amounts of appropriate fluids, and continued feeding [22]. Treatment of diarrhea with ORS is a simple, proven, high-impact intervention that can be provided in home settings by caretakers or by health care providers at community and facility levels to prevent dehydration due to diarrhea and decrease related deaths. There is evidence that ORS may reduce diarrhea specific mortality by up to 93 % [15]. However, data analysis from recent population-based household surveys show that population coverage for this basic but effective intervention is still very low, particularly in countries that are hardest hit by diarrheal diseases. In sub-Saharan Africa, only about one in three children experiencing diarrheal episodes receives ORS, and the proportion receiving zinc is below 5 % [19].

Although appropriate treatment of diarrhea is simple and can be done at home, seeking care from appropriate providers outside the home is recommended because harmful practices based on beliefs and misconceptions are prevalent, especially in low income countries where the diarrhea mortality is high. A systematic review of harmful practices in childhood diarrhea management found high and variable levels of harmful practices [3], such restriction of food and fluids, including breastfeeding. A recent analysis in six African countries found a high prevalence of fluid curtailment during episodes of diarrhea, and an association between seeking care outside of the home and higher rates of fluid curtailment, particularly for careseeking from non-government health providers [16]. Using an expanded set of countries, the current analysis investigates these findings further by assessing the prevalence of diarrhea management practices as defined in the 2004 WHO/UNICEF recommendations and their association with the source of care.

Recent studies have suggested that training public-sector providers to treat diarrhea in children with low-osmolarity ORS and zinc is effective in improving the quality of care [8]. But ensuring high and sustained implementation of appropriate treatment will require major investments in health worker training, supervision and other incentives to support correct health worker performance, as well as strategies to ensure the continuous availability of essential commodities such as ORS and zinc. Integrated community case management (iCCM) has been a pivotal strategy to reach vulnerable children and increase their chances of receiving appropriate care when sick with diarrhea or other pervasive illnesses like pneumonia and malaria.

This work was supported by [5] for Maternal, Newborn and Child Survival (“Countdown”) with the goal of generating new information useful in increasing the effectiveness of programs aimed at reducing child deaths from diarrhea. Countdown is a global initiative that tracks progress in achieving high, sustained and equitable coverage for interventions of proven effectiveness in preventing unnecessary deaths among women and children in 75 priority countries [5].

## Methods

### Data

We selected twelve countries based on the following criteria: 1) being in sub-Saharan Africa given that it is the region with the greatest proportion of diarrhea deaths; 2) being high-burden: over 10 % of country’s deaths among children 1–59 months caused by diarrhea; and 3) having recent population-based survey data available (2010 or later) with sufficient sample size for analysis. We reviewed available nationally representative population data for countries meeting the above criteria from Demographic and Health Surveys (DHS) and Multiple Indicator Cluster Survey (MICS), but retained only DHS surveys because until 2013, MICS did not collect data on care seeking for childhood diarrhea which was a key variable for this analysis [20].

The 12 countries included in the analysis are: Burkina Faso (year of survey: 2010; % deaths among 1–59 month-old caused by diarrhea in 2013: 14 %), Burundi (2010; 18 %), Cameroon (2011; 16 %), Cote d’Ivoire (2011–12; 15 %), Democratic Republic of the Congo (DRC) (2013–14; 15 %), Ethiopia (2011; 16 %), Mali (2012–13; 16 %), Niger (2012; 16 %), Nigeria (2013; 14 %), Sierra Leone (2013; 18 %), United Republic of Tanzania (2010; 12 %), and Uganda (2011; 12 %) [7, 21]. Together these countries accounted for about one-third of all under-five deaths worldwide due to diarrhea in 2013 and about two-thirds (62 %) in sub-Saharan Africa [21]. Table 4 in the Appendix presents information about the evolution of the adoption and implementation of the low-osmolarity and zinc policy in sub-Saharan African countries as well as the number and percentage of childhood deaths caused by diarrhea.

DHS collects data on childhood diarrhea treatment from nationally representative samples. In the surveys, mothers are asked if their children under five had diarrhea in the past 2 weeks. If the answer is positive, they are asked follow-up questions about care seeking and treatment, including the four recommended management interventions (ORS, zinc, increased fluids, continued feeing) as well as other potentially harmful practices including antimotility drugs.

### Analysis

We classified the quality of diarrhea management practice as good, fair, or poor based on the [22] guidelines (Table 1). We consulted with the Ministry of Health in each country to categorize the reported sources of care as facility, community based, traditional, or no care outside the home. Facility care refers to care sought from health facilities, whether public or private. Community-based care relates to care sought from community health workers, mobile clinics, village health posts, government dispensaries or health centers and health posts located at the community level, as well as pharmacies. Traditional sources of care include traditional healers, traditional practitioners as well as shops, stores, informal drug sellers and markets (Appendix Table 5). No care outside the home refers to children who were treated at home for diarrhea but for whom care was not sought outside the home.

**Table 1:** Classification of diarrhea management in children under-five into good, fair and poor based on WHO/UNICEF recommendations

Classification	Child given ORS or ORS or Zinc	Child given Increased Fluids (IF)	Child Continued Feeding (CF)
Good	Yes	Yes	Yes
Good	Yes	Yes	No
Good	Yes	No	Yes
Fair	Yes	No	No
Fair^a^	No	Yes	Yes
Fair^a^	No	Yes	No
Poor	No	No	Yes
Poor	No	No	No

^**a**^For children 6 months old and younger, defined as “good” practice

‘Good’ diarrhea management is the main outcome of interest in this analysis, and source of care is the main independent variable. We first described prevalence of diarrhea management practices across countries, then examined the country specific unadjusted association between ‘good’ diarrhea management and type of care. We finally fitted logistic regression models of ‘good’ diarrhea management practice on source of care for all countries, adjusting for the following known confounders as described below. Table 6 in the Appendix presents the estimated regression coefficients (log odds ratios for adjusted factors) from logistic regression models for the factors from Anderson’s conceptual framework, for the probability of children under five receiving good diarrhea management.

We used Andersen’s conceptual framework of access to medical care to help identify variables to control for in the regression model [1]. We identified these factors based on three main categories outlined in the Andersen’ framework. The *predisposing characteristics* included child age, mother’s age, child gender, mother’s marital status and education, partner's education, parity, number of children under five living in the household; the *enabling resources* included wealth quintile, rural or urban location, distance from health care reported by the mother as a problem in receiving health care, mother’s participation in decision making, household improved water access, open defecation and the *need characteristics* included whether there was blood in the child’s stool, as a measure of severity. However, all reported cases of diarrhea were included in the analysis and having had ‘blood in stool’ was not used for classification of diarrhoea but instead as a variable in the final regression model, thus avoiding potential misclassification issues. We assessed multicollinearity in these independent variables and retained only one of two or more variables that were highly correlated. The final model reported here includes adjustment for the following variables or potential confounders: child age, mother’s age, child gender, mother’s marital status and education, number of children under five living in household, wealth quintile, rural or urban location, if distance is a problem in receiving health care, mother’s participation in decision making, whether household has improved water, and whether there was blood in the child’s stool. These variables were all of the ones included in the initial Andersen’s model, except for mother’s participation in decision making and open defecation which were highly correlated with other variables and therefore not included in the final model. All regression analysis took into account the survey complex multi-stage sample design and sample weights. We used Stata 13 for analysis.

## Results

Table 2 presents the proportion of children with diarrhea who were reported by their mothers to have been given any of the four recommended management interventions, as well as those who were reported to have been given both ORS and zinc. The number of household and women surveyed and response rates by country are presented in Table 7 in the Appendix. The results vary widely across countries. For example, coverage of ORS ranges from 17 % in Cameroon and Cote d’Ivoire to 85 % in Sierra Leone (median = 38 %). Across countries, coverage of zinc is extremely low (due to on-going roll-out of the policy for zinc in these countries), ranging from 0 % in five out of the 12 countries to 10 % in Niger (median = 2 %). The proportion of children who were reported to have been given increased fluids during diarrhea ranges from 10 % in Nigeria to 56 % in Cameroon (median = 25 %),and the proportion for whom mothers reported continued feeding the child during the diarrhea episode ranges from 60 % in Ethiopia to 80 % in Cameroon (median = 72 %). There are no systematic patterns suggesting any pairwise association between coverages of ORS, increased fluid and continued feeding.

**Table 2:** Percent of children with diarrhea in the 2 weeks prior to the survey by type of care reported by mothers and country

Country	Weighted number of Children	Weighted # children with diarrhea	Percentage of children with diarrhea in the last 2 weeks who were given				
			ORS % (95 %CI)	ORS & Zinc % (95 %CI)	Zinc % (95 %CI)	Increased Fluids % (95 %CI)	Continued Feeding % (95 %CI)
Burkina Faso	14,001	2,064	21 (19, 24)	0 (0, 0)	0 (0, 1)	26 (23, 29)	79 (77, 82)
Burundi	7,418	1,855	38 (35, 41)	0 (0, 0)	0 (0, 0)	40 (37, 43)	72 (70, 75)
Cameroon	10,718	2,243	17 (15, 20)	0 (0, 0)	0 (0, 0)	56 (52, 59)	80 (77, 82)
Cote d’Ivoire	6,862	1,228	17 (14, 20)	0 (0, 0)	0 (0, 0)	39 (35, 42)	79 (76, 82)
DR Congo	16,968	2,852	39 (36, 42)	2 (1, 2)	2 (2, 3)	32 (29, 36)	71 (68, 75)
Ethiopia	11,042	1,483	26 (23, 30)	0 (0, 0)	0 (0, 0)	16 (12, 19)	60 (56, 65)
Mali	9,655	832	37 (32, 42)	1 (1, 2)	2 (1, 3)	14 (11, 17)	69 (65, 73)
Niger	12,268	1,734	44 (41, 47)	8 (7, 10)	10 (8, 12)	24 (21, 28)	73 (70, 77)
Nigeria	28,950	2,966	34 (31, 37)	1 (1, 2)	2 (2, 3)	10 (9, 12)	68 (65, 71)
Sierra Leone	10,814	1,201	85 (83, 87)	3 (2, 5)	4 (3, 5)	32 (27, 37)	64 (61, 68)
Tanzania	7,667	1,109	44 (40, 48)	3 (2, 4)	5 (3, 6)	18 (15, 21)	78 (75, 82)
Uganda	7,535	1,766	44 (40, 47)	1 (1, 2)	2 (1, 3)	18 (16, 21)	65 (62, 67)
Median	10,766	1,750	38 (35, 41)	1 (1, 2)	2 (1, 3)	25 (21, 29)	72 (70, 75)

Figure 1 presents the distribution of good, fair and poor diarrhea management practice by country. In 11 of the 12 countries, the prevalence of good diarrhea management practice was low, ranging from 17 % in Cote d’Ivoire to 38 % in Niger and Tanzania (median = 30 %). In Sierra Leone, the prevalence of good practice was 67 %. In contrast, levels of ‘poor’ diarrhea management are strikingly high across these countries with the exception of Sierra Leone (10 %), with a prevalence of over 50 % in 5 countries and ranging from 38 % in Cameroon to 63 % in Ethiopia (median = 48 %).

**Fig. 1:** Proportion of children under five with diarrhea in the 2 weeks prior to the survey by type of diarrhea management practice (good, fair or poor)

Figure 2 and Table 8 in the Appendix present the result on the quality of diarrhea management by source of care. In all countries except Sierra Leone, mothers of children for whom care was sought outside the home were significantly more likely to report good diarrhea management than those for whom no care was sought outside the home. However, even among children with diarrhea taken to a health facility or community provider for care, the prevalence of ‘good’ management was low (median = 52 %, range 34 % in Uganda to 64 % in Sierra Leone). For those seen at the community level, the median prevalence of good management was 40 % [range: 17 % in Burundi to 72 % in Sierra Leone], while for those taken to traditional care providers the median for good practice was 16 % [range 6 % in Burkina Faso to 67 % in Sierra Leone]. In contrast, there is substantial ‘poor’ practice even for those taken to health facility or community care with a median prevalence of 28 % and 36 % for the two sources of care respectively.

**Fig. 2:** Proportion of children under five with diarrhea in the 2 weeks prior to the survey by type of diarrhea management practice (good, fair or poor) and by source of care

Table 3 presents the adjusted odd-ratios of good diarrhea management practice by source of care. In general, as observed at bivariate level above, it suggests that sick children who were taken to health facility or community care were more likely to have had ‘good’ diarrhea management than children who were taken to traditional sources of care or not taken for care outside the home. In 11 of the 12 countries included in the analysis, mothers of children with diarrhea taken to health facility were 3.3 to 17 times more likely to have reported ‘good’ management for their condition than mothers of children not taken outside the home for care, after adjusting for selected confounders. This range was 1.4 to 13 for community care for the 12 countries. The exception is Sierra Leone, where ‘good’ management of diarrhea is high (over 60 %) regardless of place of care (Table 7 in the Appendix). In 4 countries, (Burkina Faso, Cote d’Ivoire, Nigeria, Sierra Leone) children taken for care to traditional providers are less likely to have ‘good’ management for their condition than children not taken anywhere for care. There is no statistically significant difference between traditional care and no care, except in Nigeria, where traditional care is more detrimental to children than no care. Table 3 presents the adjusted odds ratios and 95 % confidence intervals for ‘good’ diarrhea management, and Table 9 in the Appendix present the unadjusted estimates.

**Table 3:** Adjusted odds ratios and 95 % confidence intervals for good diarrhea management for enabling, predisposing, and need related factors per Anderson’s model*

	Adjusted odds ratio and 95 % confidence interval for good management (Reference: no care outside the home)		
	Facility Care	Community Care	Traditional Care
Burkina Faso	12.0 (8.0, 18.2)*	5.7 (4.0, 8.2)*	0.7 (0.3, 1.8)
Burundi	11.2 (8.3, 15.1)*	2.2 (0.9, 5.3)	2.6 (0.9, 7.8)
Cameroon	17.0 (10.9, 26.7)*	8.4 (5.6, 12.6)*	1.1 (0.7, 1.8)
Cote d’Ivoire	9.6 (5.7, 16.3)*	9.0 (4.1, 19.9)*	0.7 (0.3, 1.5)
DR Congo	6.0 (4.5, 8.0)*	2.7 (2, 3.8)*	1.6 (0.8, 3.4)
Ethiopia	9.5 (6.1, 14.9)*	5.9 (3.1, 11.4)*	1.5 (0.2, 9.9)
Mali	10.3 (4.7, 22.6)*	6.5 (3.9, 10.9)*	1.6 (0.9, 2.8)
Niger	5.2 (2.5, 11.0)*	13.0 (9.4, 18.2)*	1.4 (0.8, 2.5)
Nigeria	4.4 (3.2, 6.2)*	3.8 (2.2, 6.5)*	0.8 (0.4, 1.6)*
Sierra Leone	0.9 (0.7, 1.4)	1.4 (0.9, 2.3)	0.9 (0.3, 3.1)
Tanzania	7.1 (3.7, 13.6)*	5.1 (3.2, 8.1)*	
Uganda	3.3 (2.2, 4.9)*	6.5 (4.2, 10.1)*	1.8 (0.7, 4.7)

*Significantly different from 1 with p < 0.05

*The final model measuring the probability of ‘good’ diarrhea management on source of care was adjusted by the following variables

• predisposing characteristics -child’s age, mother’s age, child’s gender, mother’s marital status and education, number of children under five living in household

• enabling resources- wealth quintile, rural or urban location, if distance is a problem in receiving health care, participating in decision making, household improved water access

• need characteristic -whether there was blood in the child’s stool

A test for the interaction between child age and place of care indicates that the association between good diarrhea management and place of care was significantly less pronounced among children aged 0 to 5 months in seven of these eleven countries (Burkina Faso, Burundi, Cameroon, Cote d’Ivoire, DR Congo, Mali and Niger) than it is among older children. That is, older children with diarrhea taken to a health facility for care were given higher quality care than those who were not taken outside the home for care, but younger children taken to health facility were only slightly better managed than those with no care in these seven countries. However, children aged 0 to 5 months who were taken to health facility for care had good diarrhea management more often than those with no care (Table 10 in the Appendix).

The adjusted effects of community care versus facility care on the probability of receiving good diarrhea management are shown in Fig. 3. Careseeking from health facilities does not appear to result systematically in higher likelihood of good diarrhea management than care from community providers. In two countries (Niger and Uganda), community care was of higher quality than facility care, and in four countries (Burkina Faso, Burundi, Cameroon and DR Congo) management for those with community care is lower than facility care. In the remaining six, there is no statistically significant difference in the quality of diarrhea management between these two sources of care.

**Fig. 3:** Adjusted odds ratio of good diarrhea management, for those who were taken to community-based care, compared to those who were taken to health facilities for care. Note to Fig. 3 text: If odds ratios and confidence intervals are higher than 1, the average management for those who sought community care was superior to those who sought facility care. If odds ratios and confidence intervals are lower than 1, the average management for those who sought community care was inferior to those who sought facility care

## Discussion

Diarrhea remains a high burden disease despite the availability of simple, affordable, and effective treatments. Recent studies have shown high levels of harmful practices during childhood diarrhea, including the curtailment of fluids and food during illness episodes [3, 13, 16, 17, 23]. This analysis assesses the quality of diarrhea management by source of care in twelve sub-Saharan African countries in which diarrhea is a major cause of under-five deaths. Based on mothers’ reports of the treatment given to their children during episodes of diarrhea in the 2 weeks preceding the survey, we categorized diarrhea management practice as good, fair or poor based on WHO/UNICEF recommendations. We then assessed the association between ‘good’ diarrhea management practice and the source of care, distinguishing between care from health facilities, community care, traditional care and no care outside the home. The results indicate that few children are given high quality care for diarrhea in 11 of the 12 countries (range 17 % to 38 % with a median of 27 %). Particularly striking is the pervasiveness and high levels of poor diarrhea management, ranging from 38 % to 63 % with a median of 49 %. Of the 12 countries, Sierra Leone is the exception with the highest level of good management: about two-thirds of children (67 %) with diarrhea provided with good management and only about 10 % of children provided with ‘poor’ management.

Low levels of coverage of ORS is a major driver of poor diarrhea quality care. Except in Sierra Leone, where ORS coverage in 2013 was 85 % -and has been consistently over 50 % since at least 2005-, coverage of ORS was below 50 % in all countries, and was only 17 % in Cote d’Ivoire and Cameroon.

Why is the quality of diarrhea management so much better in Sierra Leone than in the other 11 countries studied? We explored possible reasons, keeping in mind that challenges to the health systems associated with the recent Ebola epidemic have had a negative impact on child health care since 2013 [18]. Sierra Leone’s success in scaling up basic child health interventions, including ORS, has been attributed to several important contextual factors [24, 6, 25], including the opportunity to rebuild the health system after the 11-year civil war that ravaged the country between 1999 and 2002 and displaced as many as 2 million out of the 5.5 million population. The war also took a particular toll of the country’s health infrastructure [23, 24]. During these years, a large proportion of the population lived in internally displaced population camps. In camps, cholera outbreaks were not uncommon and were mostly managed with ORS largely distributed by community volunteers referred to as “Blue Flag Volunteers”. ORS was widely accessible and available in attractive orange-flavor low-osmolarity formulation. Following the civil war, nationwide efforts were made to ensure that the supply chain was maintained at each level [23]. Deployment of community health volunteers was also associated with a reduced treatment burden at facilities and less reliance on traditional treatments [25]. As part of this transformation, in April 2010 the government of Sierra Leone abolished healthcare costs for pregnant women, new mothers and children under five. As a result, many more pregnant women, new mothers and their young children are now coming to health centers [10]. The particular case of Sierra Leone shows that through strong government support and local efforts, important health intervention can be scaled up in a sustained manner.

Across countries, our analysis further showed that children with diarrhea for whom care was sought from health facilities or community health providers were more likely to receive good management than those for whom care was sought from traditional or informal sources or those for whom no care was sought. Thus, although treatment of diarrhea is simple and can be managed at home with appropriate knowledge and supplies, it is essential to continue to recommend that children with diarrhea seek appropriate care from facilities or health community services. This recommendation must be accompanied by significant improvement in quality of care at health facilities and community health providers. Poor quality of care at health facilities and community health workers represents an enormous missed opportunity to prevent unnecessary child deaths due to diarrhea.

The comparisons by type of provider revealed that in six of the countries, children for whom care was sought from community-based health providers are equally likely to have been given ’good’ management as those for whom care was sought from health facilities. This, further corroborates studies of quality of care provided by community health workers that demonstrated that this health *cadre* can provide treatment services of the same quality as health facilities [11, 14].

There are limitations in our analysis that should be considered when interpreting the findings. Our measure of diarrhea management practice was based mother’s recall of care provided to the child during episode of diarrhea. This could have led to differential recall bias and may not entirely reflect the level of quality of care in facilities or from community-based workers. For instance, mothers are more likely to recall ORS than, other treatments like zinc, which might be misremembered as an antibiotic or other medication. The growing body of research on the validity of mothers’ reports of child survival interventions has also raised important issues that are likely to apply here [2] and could only be addressed through carefully designed validation studies. We were also unable to assess the severity of the diarrhea, which may affect mother’s decisions about careseeking as well as the type of management received at the health facility. Further studies are needed to explore the role of local and cultural beliefs and practices in determining caregiver understandings of diarrhea and appropriate responses are also important, and will require further study using qualitative methodologies [4].

## Conclusions

Despite these limitations, the findings presented in this paper show clearly that there is an important missed opportunity to prevent child deaths due to diarrhea by making sure that health care providers are managing childhood diarrhea appropriately, including advising caregivers effectively about providing ‘good’ diarrhea management at home and the importance of seeking care outside the home. Although there is variation across countries, the results also suggest that community-based providers can provide access to management at levels of quality comparable to that provided at health facilities, lending support to advocates of more widespread implementation of iCCM strategies.

## Figures and Tables

**Table 5:** Classification of sources of care for child diarrhea in countries included in the analysis (categories are those included in the DHS data used in the analysis)

Classification of country specific sources of care was done exclusively for this analysis and as determined by country and by the specific health systems in place. Ministries of Health in each countries were consulted for this classification

Facility

Community

Traditional/ informal

**Table 6:** Adjusted coefficients (log odds ratios) from logistic regression models of good diarrhea management adjusting for factors from Anderson’s conceptual framework. Associations that are significantly different from zero at *p* = 0.05 are shown in red

## Appendix

**Table 4:** Estimates on diarrhea specific mortality among children under five and evolution of the adoption and implementation of the national policy on low-osmolarity ORS and zinc for management of diarrhea - Sub-Saharan African countries

	2015 estimates		Status of policy on low osmolarity ORS and zinc for management of diarrhea		
Country	Total n. under five deaths due to diarrhea	% deaths among children 1–59 months caused by diarrhea	2008	2010	2015
Angola	24,927	21 %	No	Partial	Yes
Benin	3,996	16 %	Yes	Yes	Yes
Botswana	157	13 %	Partial	Yes	Yes
Burkina Faso^a^	4,975	12 %	Yes	Yes	Yes
Burundi^a^	3,716	15 %	Partial	Partial	Yes
Cabo Verde	14	10 %	-	-	-
Cameroon	8,032	16 %	Yes	Yes	Yes
Central African Republic	2,194	15 %	-	No	No
Chad	11,360	19 %	Yes	Yes	Yes
Comoros	142	13 %	-	-	Yes
Congo	519	12 %	Yes	Yes	Yes
Côte d’Ivoire^a^	5,697	13 %	Partial	Partial	Yes
Democratic Republic of the Congo^a^	32,047	15 %	Yes	Yes	Yes
Djibouti	116	16 %	-	Yes	Yes
Equatorial Guinea	200	11 %	Yes	Yes	Yes
Eritrea	694	14 %	Partial	Partial	Yes
Ethiopia^a^	15,535	15 %	Yes	Yes	Yes
Gabon	160	11 %	Yes	Yes	Yes
Gambia	487	16 %	-	No	Yes
Ghana	3,657	12 %	Partial	Yes	Yes
Guinea	3,506	12 %	Yes	No	Yes
Guinea-Bissau	562	17 %	No	Partial	Yes
Kenya	5,442	13 %	Yes	Yes	Yes
Lesotho	541	15 %	Yes	Partial	Yes
Liberia	937	13 %	Partial	Yes	Yes
Madagascar	3,665	15 %	Yes	Yes	Yes
Malawi	3,062	11 %	Partial	Yes	Yes
Mali^a^	7,807	14 %	Partial	Partial	Yes
Mauritania	1,186	18 %	No	No	-
Mauritius	5	6 %	-	-	-
Mozambique	7,341	13 %	Partial	Partial	Yes
Namibia	299	14 %	-	-	-
Niger^a^	9,873	16 %	Yes	Yes	Yes
Nigeria^a^	76,980	15 %	Yes	Yes	Yes
Rwanda	1,033	13 %	Yes	Yes	Yes
Sao Tome and Principe	23	12 %	-	-	Yes
Senegal	2,403	16 %	Yes	Yes	Yes
Seychelles	0	2 %	-	-	-
Sierra Leone^a^	2,784	15 %	Partial	Yes	Yes
Somalia	8,759	20 %	-	Partial	Yes
South Africa	3,627	12 %	Yes	Yes	Yes
South Sudan	3,243	14 %	-	-	No
Sudan	9,536	18 %	Yes	Yes	Yes
Swaziland	230	13 %	-	Yes	Yes
Togo	1,636	13 %	Yes	Yes	Yes
Uganda^a^	7,001	12 %	Yes	Yes	Yes
United Republic of Tanzania^a^	8,000	13 %	Yes	Yes	Yes
Zambia	3,469	13 %	Yes	Yes	Yes
Zimbabwe	3,677	14 %	Yes	Yes	Yes

Notes:

Indicator: Low-osmolarity oral rehydration salts and zinc for management of diarrhea

Definition: National policy on management of diarrhoea with low-osmolarity oral rehydration salts and zinc has been adopted and implemented

Criteria for ranking

Yes: national policy or guidelines adopted on use of low-osmolarity oral rehydration salts and zinc for management of diarrhoea

No: no national policy or guidelines adopted on the use of low-osmolarity oral rehydration salts and zinc for managements of diarrhoea

Partial: National policy or guidelines adopted on use of low osmolarity ORS and zinc for management of diarrhoea but no implementation; OR no national policy or guidelines adopted but implementation in selected areas; OR national policy or guidelines adopted and/or implementation commenced for either low osmolarity ORS or zinc use, but not for both

Source: Mortality estimates from WHO-MCEE estimates of child cause of death, 2000–2015 and policy data from WHO Global Maternal Newborn Child and Adolescent Health Policy Indicator Survey by the World Health Organization Department of Maternal Child Adolescent Health

^a^ Countries included in the analysis

**Table 7:** Number of household and women surveyed and response rates by country

Country	Survey Year	Household (N)	Women 15–49 years old (N)	Response rate for women (%)
Burkina Faso	2010	8,619	10,364	98.4
Burundi	2010	4,807	4,916	95.5
Cameroon	2011	6,537	7,655	96.4
Cote d’Ivoire	2011	4,553	5,431	91.0
DR Congo	2013	10,428	11,293	98.5
Ethiopia	2011	7,534	7,764	93.2
Mali	2012	5,982	6,723	94.4
Niger	2012	6,673	7,680	93.5
Nigeria	2013	17,723	20,192	96.7
Sierra Leone	2013	7,263	8,524	96.5
Tanzania	2010	4,907	5,358	95.2
Uganda	2011	4,618	4,909	89.4

**Table 8:** Percent of children under five with diarrhea in the 2 weeks prior to the survey by type of diarrhea management practice (good, fair or poor) and provider

	Careseeking for Diarrhea^a^											
	Facility Care			Community Care			Traditional Care			No Care outside the home		
	Good Practice	Fair Practice	Poor Practice	Good Practice	Fair Practice	Poor Practice	Good Practice	Fair Practice	Poor Practice	Good Practice	Fair Practice	Poor Practice
Burkina Faso	47 %	24 %	29 %	28 %	19 %	53 %	5 %	24 %	72 %	6 %	20 %	74 %
Burundi	51 %	23 %	26 %	17 %	40 %	43 %	17 %	13 %	70 %	9 %	28 %	63 %
Cameroon	59 %	27 %	14 %	40 %	39 %	21 %	8 %	45 %	47 %	8 %	47 %	46 %
Cote d’Ivoire	42 %	26 %	32 %	40 %	24 %	36 %	5 %	28 %	67 %	8 %	34 %	58 %
DR Congo	56 %	21 %	22 %	37 %	24 %	38 %	24 %	21 %	55 %	19 %	22 %	59 %
Ethiopia	42 %	31 %	27 %	33 %	25 %	42 %	10 %	21 %	69 %	7 %	12 %	81 %
Mali	61 %	21 %	18 %	50 %	24 %	26 %	21 %	18 %	61 %	15 %	19 %	66 %
Niger	52 %	19 %	29 %	63 %	22 %	16 %	16 %	17 %	67 %	12 %	18 %	70 %
Nigeria	37 %	19 %	44 %	32 %	23 %	45 %	6 %	10 %	83 %	12 %	10 %	79 %
Sierra Leone	64 %	28 %	8 %	72 %	23 %	6 %	67 %	17 %	16 %	68 %	17 %	16 %
Tanzania	56 %	10 %	33 %	49 %	16 %	35 %	--	--	--	16 %	9 %	75 %
Uganda	34 %	21 %	45 %	49 %	25 %	26 %	19 %	18 %	63 %	13 %	14 %	73 %

^a^A test for difference in diarrhea management practice for different provider type is highly significant in each of these twelve surveys. This was an overall test of association, indicating that the average diarrhea management is different by source of care

**Table 9:** Unadjusted odds ratios and 95 % confidence intervals for ‘good’ diarrhea management

Unadjusted odds ratio and 95 % confidence interval for good management (Reference: no care outside the home)			
	Facility Care	Community Care	Traditional Care
Burkina Faso	13.8 (9.2, 20.8)*	6 (4.2, 8.4)*	0.7 (0.3, 1.8)
Burundi	10.9 (8.2, 14.5)*	2.2 (0.9, 5.7)	2.2 (0.7, 6.7)
Cameroon	17.4 (11.7, 25.9)*	7.9 (5.4, 11.6)*	1.0 (0.6, 1.6)
Cote d’Ivoire	8.4 (5, 14.3)*	7.7 (3.6, 16.4)*	0.6 (0.3, 1.4)
DR Congo	5.4 (4.1, 7.1)*	2.6 (1.9, 3.5)*	1.4 (0.7, 2.9)
Ethiopia	9.3 (6, 14.2)*	6.3 (3.2, 12.3)*	1.4 (0.2, 12.2)
Mali	9.2 (4.5, 18.9)*	5.8 (3.5, 9.6)*	1.6 (0.9, 2.8)
Niger	8 (3.5, 17.9)*	12.1 (8.8, 16.6)*	1.4 (0.8, 2.4)
Nigeria	4.4 (3.1, 6.1)*	3.5 (2.0, 5.9)*	0.5 (0.3, 1.0)*
Sierra Leone	0.9 (0.6, 1.3)	1.3 (0.8, 2.1)	1.0 (0.3, 3.4)
Tanzania	7.1 (3.8, 13.4)*	5.2 (3.3, 8.4)*	
Uganda	3.6 (2.4, 5.2)*	6.6 (4.4, 10.1)*	1.7 (0.6, 4.4)

***Significantly different from 1 with *p* < 0.05

**Table 10:** Crude odds ratios and 95 % confidence intervals for good diarrhea management among children age 0 to 5 months

	Crude odds ratio and 95 % confidence interval for good management among children age 0–5 months (Reference: no care outside the home)		
	Facility Care	Community Care	Traditional Care
Burkina Faso	2.1 (0.6, 7.4)	0.8 (0.3, 2.6)	0.3 (0.1, 1.6)
Burundi	1.2 (0.5, 2.9)	NE	NE
Cameroon	5.8 (1.1, 31.8)*	2.2 (0.7, 6.8)	0.9 (0.2, 3.7)
Cote d’Ivoire	1.1 (0.3, 4.3)	0.6 (0.1, 4)	0.4 (0.1, 2.7)
DR Congo	2.9 (1.1, 7.5)*	1.5 (0.7, 3.3)	5 (1.3, 19.3)*
Ethiopia	8.4 (1.9, 37.7)*	6.7 (0.9, 47.9)	NE
Mali	1.1 (0.1, 12.1)	9.7 (2.4, 38.4)*	0.9 (0.2, 4.2)
Niger	NE	4.3 (2, 9.1)*	1.7 (0.5, 6.6)
Nigeria	8.1 (2.2, 29.4)*	12.7 (2.5, 63.7)*	1.2 (0.1, 11.1)
Sierra Leone	3.4 (1.1, 10.7)*	51.4 (4.6, 571.3)*	NE
Tanzania	0.5 (0, 6.1)	3.1 (0.9, 11.3)	NE
Uganda	1.2 (0.4, 3.5)	1.8 (0.7, 5)	NE

NE, not estimable

***Significantly different from 1 with *p* < 0.05

## Abbreviations

DHS: Demographic and Health Survey
DRC: Democratic Republic of the Congo
MICS: Multiple Indicator Cluster Surveys
ORS: Oral Rehydration Salts
UNICEF: United Nations Children’s Fund
WHO: World Health Organization
